This article has been retracted.

# Evidence-Based Analysis on Observation for Nursing Care of Patients with Intra-Aortic Balloon Pumping

**DOI:** 10.1155/2021/5954343

**Published:** 2021-08-26

**Authors:** Yan Zhang, Huali Chen, Lihua Li, Zhaofen Zheng, Jianqiang Peng, Juan Zhou, Xiaoying Qiu, Fang Li

**Affiliations:** ^1^Department of Cardiovascular Internal Medicine, Clinical Medical Research Center of Heart Failure, Hunan Provincial People's Hospital (The First Affiliated Hospital of Hunan Normal University), Changsha 410005, China; ^2^Clinical Medical Research Center of Heart Failure, Hunan Provincial People's Hospital (The First Affiliated Hospital of Hunan Normal University), Changsha 410005, China; ^3^Quality Control Office of Nursing Department, Hunan Provincial People's Hospital (The First Affiliated Hospital of Hunan Normal University), Changsha 410005, China; ^4^Hunan Province Disinfection Supply Quality Control Center, Changsha 410005, China; ^5^First Department, Disinfection Supply Center, Hunan Provincial People's Hospital (The First Affiliated Hospital of Hunan Normal University), Changsha 410005, China; ^6^Department of Hematology, Hunan Provincial People's Hospital (The First Affiliated Hospital of Hunan Normal University), Changsha 410005, China

## Abstract

In this study, data analysis was performed on 52 patients. According to the different outcomes and discharge diagnosis of patients, data on sedative use, emotions, behavioral abnormalities, hearing loss, pain, total time on board the IABP (intra-aortic balloon pumping), and days of hospitalization of patients were collected. The data were subjected to frequency analysis, paired chi-square analysis, chi-square test, Poisson regression analysis, and stepwise regression analysis. Some findings of the analysis included the following: Between outcome and admission diagnosis, the analysis showed that significant differences existed between paired data. Patients with heart failure and acute myocardial infarction are in an unhealed state, and most patients with coronary atherosclerotic heart disease, myocarditis, and heart disease showed improvement. The samples taken by different sedatives showed no significant differences in the emotional and behavioral abnormalities, hearing loss, and pain. A total of 1 item of hospital stay had a significant negative impact on the total operation time of IABP. However, discharge diagnosis and admission diagnosis did not affect the total time on board the IABP. The dorsalis pedis artery pulse condition has a significant negative effect on the total time on board the IABP.

## 1. Introduction

Intra-aortic balloon pumping (IABP) [1] is a technique where a balloon and catheter are put into the artery from the femoral artery while a counterpulsation machine is connected outside the body and the patient's blood pressure or electrocardiogram (ECG) signal is used for the control. The balloon deflates before the heart contracts, leading to increase of cardiac output. Subsequently, the balloon inflates during diastole. Based on a large volume of reported evidence, IABP has been an important means to rescue critically ill patients with syndromes such as heart failure, cardiogenic shock, and low cardiac output [2–5].

As reported by Ansari and Garcia [6], when used in ischemic and nonischemic patients, IABP is associated with fewer clinical complications. Ansari and Garcia [6] also found that different mechanical support devices can be used for cardiogenic shock and may provide different results. Using chest X-ray and CT, Lara-Breitinger et al. [7] indicate that the movement of the distal end of IABP in armpits may lead to accidental occlusion of shape-memory alloy and intestinal ischemia. Bhimaraj et al. [8] show that percutaneous axillary IABP implantation is a method for prolonging the mechanical circulatory support in patients with advanced heart failure. In a case report, Goteti et al. [9] demonstrate the importance of early insertion of IABP in complex cases of acute heart failure. In another case reported by Al-Ani et al. [10], the hemostasis technique of arteriotomy can be used for axillary intra-aortic balloon pumping in dysfunctional patients.

The above observations indicate that the nursing care of patients with IABP is important for clinical cases [11]. In this work, we have analyzed the nursing care of patients with IABP for the following observations. Data analysis was performed on 52 patients. According to the different outcomes and discharge diagnosis of patients, data on sedative use, emotion, behavioral abnormalities, hearing loss, pain, total time on board the IABP, and days of hospitalization of patients were collected. The data were subjected to frequency analysis, paired chi-square analysis, chi-square test, Poisson regression analysis, and stepwise regression analysis. The work may support many IABP analyzing works [12], since the mathematic analysis is important for clinical and biochemical studies [13–16].

## 2. Objective and Methods

Table 1 shows the frequency analysis results of 52 patients. The raw information is shown in the supplementary file (available here). The results are analyzed using SPSS (Statistical Product and Service Solutions). Table 1 shows that “males” are relatively more in the samples from the perspective of gender, with the proportion of 73.08%. From the distribution of outcomes, the majority of samples were “improved,” and the proportion was 57.69%. “Acute myocardial infarction” was selected in 51.92% of the samples.

## 3. Results and Discussion

As shown in Table 2, the paired chi-square test was used to study the paired difference relationship between admission diagnosis and outcomes. The number of paired comparison categories in this study was greater than 2 (i.e., paired multiclassification). Hence, the Bowker test was used for this study. Significant differences between paired data at the 0.05 level (chi = 49.333, *p* ≤ 0.001) were noted. Patients with heart failure and acute myocardial infarction are in an unhealed state, and most patients with coronary atherosclerotic heart disease, myocarditis, and heart disease are improved. In summary, Bowker examined differences between study outcomes and hospital admissions and analysis revealed significant differences between paired data.

As shown in Table 3, the chi-square test (cross-analysis) was used to study the independence of the difference relationship between the use of sedatives and the total three items of emotional and behavioral disorders, hearing loss, and pain. From Table 3, it can be seen that the samples of different sedatives do not show significant differences in the three items of emotional and behavioral disorders, hearing loss, and pain (*p* > 0.05), which means that the samples of different sedatives show consistent differences in the three items of emotional and behavioral disorders, hearing loss, and pain.

As shown in Table 4, discharge diagnosis, admission diagnosis, and hospital stay were taken as independent variables. The total operation time of IABP was taken as dependent variable for Poisson regression analysis. As shown in Table 4, the model pseudo-*R* formula (McFadden *R* formula) is 0.022, which means that the discharge diagnosis, admission diagnosis, and hospital stay can explain the change of 2.2% of the total operation time of IABP. As shown in Table 4, the model formula was as follows: log (*u*) = 3.148 + 0.015^*∗*^ hospital discharge diagnosis −0.014^*∗*^ hospital admission diagnosis −0.015^*∗*^ hospital stay (where *U* represents the expected mean). The final specific analysis shows the following.

The regression coefficient value for discharge diagnosis was 0.015, but it was not significant (*z* = 1.434, *p*=0.152 > 0.05), suggesting that the discharge diagnosis did not affect the total IABP operation time.

The regression coefficient value for the admission diagnosis was −0.014, but it was not significant (*z* = −0.561, *p*=0.575 > 0.05), suggesting that the admission diagnosis did not affect the total IABP time on board.

The regression coefficient of inpatient hospital stay was −0.015, and it was significant at 0.01 level (*Z* = −2.670, *p*=0.008 < 0.01), indicating that inpatient hospital stay had a significant negative effect on the total operation time of IABP. And, an OR of 0.985 represented a 0.985-fold change in IABP's total on-board time when hospital stays were increased by one unit.

According to the summary and analysis, it can be seen that the number of hospital days has a negative impact on the total operation time of IABP. However, discharge diagnosis and admission diagnosis did not affect the total time on board the IABP, as shown in Figure 1.

As shown in Table 5, the dorsalis pedis pulse was used as the independent variable and the total time on board the IABP was used as the dependent variable for stepwise regression analysis. After automatic recognition by the model, finally the remaining one item of dorsalis pedis artery pulse was included in the model and the model formula was as follows: total time on board the IABP = 36.755–2.103^*∗*^ dorsalis pedis artery pulse. An *R*-square value of 0.150 means that the dorsalis pedis pulse explains 15.0% of the change in total time on board the IABP. Moreover, the model passed the *F* test (*F* = 8.857, *p*=0.004 < 0.05), indicating that the model was effective. In addition, the multicollinearity of the model is tested, and it was found that all the VIF values in the model are less than 5, which means that there is no collinearity problem. And, the value of D-W is near the number 2, which indicates that the model has no autocorrelation and there is no correlation between the sample data, so the model is good.

The final specific analysis showed that the regression coefficient value of the dorsalis pedis pulse was −2.103 (*t* = −2.976, *p*=0.004 < 0.01), which meant that the dorsalis pedis pulse had a significant negative effect on the total operation time of IABP.

## 4. Conclusions

In this study, data analysis was performed on 52 patients. According to the different outcomes and discharge diagnosis of patients, data on sedative use, emotions, behavioral abnormalities, hearing loss, pain, total time on board the IABP, and days of hospitalization of patients were collected. The data were subjected to frequency analysis, paired chi-square analysis, chi-square test, Poisson regression analysis, and stepwise regression analysis. Some findings of the analysis included the following: (1) Between outcome and admission diagnosis, the analysis showed that significant differences existed between paired data. Patients with heart failure and acute myocardial infarction are in an unhealed state, and most patients with coronary atherosclerotic heart disease, myocarditis, and heart disease are in the improved state. (2) The samples taken by different sedatives showed no significant differences in the emotional and behavioral abnormalities, hearing loss, and pain. (3) A total of 1 item of hospital stay had a significant negative impact on the total operation time of IABP. However, discharge diagnosis and admission diagnosis did not affect the total time on board the IABP. (4) The dorsalis pedis artery pulse condition has a significant negative effect on the total time on board the IABP.

## Figures and Tables

**Figure 1:** Regression coefficient of the independent variable to the dependent variable.

**Table 1:** Frequency analysis results (52 patients).

Name	Options	Frequency	Percentage	Cumulative percentage
Gender	Female	14	26.92	26.92
	Male	38	73.08	100.00
	Other	14	26.92	26.92

Lapse	Improve	30	57.69	84.62
	Not cured	8	15.38	100.00

Discharge diagnosis	Unstable angina pectoris	2	3.85	3.85
	Coronary atherosclerotic heart disease	8	15.38	19.23
	Heart failure (cardiac function class III or above)	1	1.92	21.15
	Cardiogenic shock	3	5.77	26.92
	Acute ST-segment elevation anterior myocardial infarction	1	1.92	28.85
	Acute inferior myocardial infarction	1	1.92	30.77
	Acute anterior myocardial infarction	2	3.85	34.62
	Acute myocardial infarction < surgical intervention > (including 1 stent)	2	3.85	38.46
	Acute myocardial infarction	27	51.92	90.38
	Septic shock	1	1.92	92.31
	Viral myocarditis	2	3.85	96.15
	Senile valvular heart disease	1	1.92	98.08
	Old inferior myocardial infarction	1	1.92	100.00

Total		52	100.0	100.0

**Table 2:** Paired chi-square analysis results (*n* = 52).

Pair	Name	Admission diagnosis						Total	*χ* ^2^	*p*
		Coronary atherosclerotic heart disease	Heart failure	Myocarditis	Heart disease	Acute myocardial infarction	Anonymous			
Lapse	Other	0	0	0	6	7	1	14	49.333	≤0.001^*∗∗*^
	Improve	4	0	1	16	8	1	30		
	Not cured	0	2	0	1	2	3	8		
	4.0	0	0	0	0	0	0	0		
	5.0	0	0	0	0	0	0	0		
	6.0	0	0	0	0	0	0	0		

Total		4	2	1	23	17	5	52		

^*∗∗*^*p* < 0.01.

**Table 3:** Chi-square test analysis results (*n* = 52).

Subject	Name	Use of sedatives (%)			Total	*χ* ^2^	*p*
		Diazepam tablets	Anonymous	Estazolam tablets			
Abnormal mood and behavior	Occasional agitation	1 (2.94)	1 (5.88)	0 (0.00)	2 (3.85)	11.995	0.847
	Loss of consciousness has occurred	0 (0.00)	1 (5.88)	0 (0.00)	1 (1.92)		
	Sleepiness	0 (0.00)	1 (5.88)	0 (0.00)	1 (1.92)		
	Anonymous	26 (76.47)	8 (47.06)	1 (100.00)	35 (67.31)		
	Coma	3 (8.82)	2 (11.76)	0 (0.00)	5 (9.62)		
	Vague, drowsy, clear	1 (2.94)	0 (0.00)	0 (0.00)	1 (1.92)		
	Dysphoria	0 (0.00)	1 (5.88)	0 (0.00)	1 (1.92)		
	Restless	2 (5.88)	2 (11.76)	0 (0.00)	4 (7.69)		
	Restless	0 (0.00)	1 (5.88)	0 (0.00)	1 (1.92)		
	Restlessness, lethargy	1 (2.94)	0 (0.00)	0 (0.00)	1 (1.92)		
Total		34	17	1	52		

Hearing loss	Anonymous	14 (41.18)	9 (52.94)	0 (0.00)	23 (44.23)	1.445	0.486
	Yes	20 (58.82)	8 (47.06)	1 (100.00)	29 (55.77)		
Total		34	17	1	52		

Pain	Anonymous	7 (20.59)	4 (23.53)	0 (0.00)	11 (21.15)	0.332	0.847
	Pain	27 (79.41)	13 (76.47)	1 (100.00)	41 (78.85)		
Total		34	17	1	52		

**Table 4:** Summary of Poisson regression analysis results (*n* = 52).

Item	Regression coefficient	Standard error	*Z* value	*p* value	OR value	OR value 95% CI
Discharge diagnosis	0.015	0.010	1.434	0.152	1.015	0.995∼1.036
Admission diagnosis	−0.014	0.025	−0.561	0.575	0.986	0.938∼1.036
Inpatient days	−0.015	0.006	−2.670	0.008	0.985	0.974∼0.996
Intercept	3.148	0.148	21.218	≤0.001	23.292	17.415∼31.154

Dependent variable: total operation time of IABP. McFadden *R* formula: 0.022.

**Table 5:** Results of stepwise regression analysis (*n* = 52).

	Nonstandardized coefficient		Normalization coefficient	*t*	*p*	VIF	*R* ^2^	Adjust *r*	*F*
	*B*	Standard error	Beta						
Constant	36.755	5.260	-	6.987	≤0.001^*∗∗*^	—	0.150	0.133	*F* (1, 50) = 8.857, *p*=0.004
Dorsalis pedis artery pulsation	−2.103	0.707	−0.388	−2.976	0.004^*∗∗*^	1.000			

Dependent variable: total operation time of IABP. D-W value: 2.019. ^*∗∗*^*p* < 0.01.

## Data Availability

All data used to support this work are included within the paper and the supplementary file.

## Supplementary Materials

Supplementary Materials The supplementary file includes raw data for the SPSS analysis.
